The article "Recent global warming as a proximate cause of deforestation and forest degradation in northern Pakistan" was retracted in 2022. Reasons: compromised peer review; a conflict of interest; concerns about the authorship.

# Recent global warming as a proximate cause of deforestation and forest degradation in northern Pakistan

**DOI:** 10.1371/journal.pone.0260607

**Published:** 2022-01-21

**Authors:** Saif Ullah, Nizami Moazzam Syed, Tian Gang, Rana Shahzad Noor, Sarir Ahmad, Muhammad Mohsin Waqas, Adnan Noor Shah, Sami Ullah

**Affiliations:** 1 College of Economics & Management, Northeast Forestry University, Harbin, China; 2 Department of Forestry & Wildlife, Management, University of Haripur, Haripur, Pakistan; 3 Department of Agriculture, Biological, Environment and Energy Engineering, College of Engineering, Northeast Agricultural University, Harbin, China; 4 Faculty of Agricultural Engineering and Technology, PMAS-Arid Agriculture University, Rawalpindi, Pakistan; 5 Department of Agricultural Engineering, Khwaja Fareed University of Engineering and Information Technology, Rahim Yar Khan, Punjab, Pakistan; 6 Department of Chemistry, College of Science, King Khalid University, Abha, Saudi Arabia; Ghazi University Dera Ghazi Khan, PAKISTAN

## Abstract

Instrumental climatological records such as weather stations data of northern areas of Pakistan are not sufficient to assess *the forest extreme events* reliably. To understand the past climatic variability, tree ring width based climatic reconstruction is the best alternative to trace climate variability that goes back in time. *Quercus Incana* is the most sensitive species to drought and climatic variation in northern Pakistan. However, very little research quantifies the rate of ongoing climatic changes. A total of 65 tree cores were collected from two sites to understand the radial growth of *Q*. *Incana* to extreme drought events. The radial growth is mainly affected by high temperatures during May-July. In addition, radial growth exhibits a positive correlation with February-June precipitation while it is negatively correlated with the September precipitation. The radial growth decrease, particularly in harsh climatic conditions. The reconstructed tree ring record was strongly coherent with the May-June self-calibrated Palmer drought severity index (scPDSI) and reliable in reconstructing drought variability for the period 1750–2014. During the past 264 years, wet periods were found during 1980–2010, 1812–1836, and 1754–1760, while dry periods were found during 1896–1922, 1864–1876, and 1784–1788. Our reconstruction explains 39.8% of the scPDSI variance. The extreme drought and wet years we arrived at were in close agreement with the drought and wet periods that occurred in northern Pakistan. Wavelet analysis revealed drought variability at periodicities of 2.2–2.5, 3.3, 3–4, 16.7, 16.8, and 68–78.8 years. Hence it is concluded that deforestation and forest degradation rate increased with extreme drought and wet years. Overall, the variation of drought in northern Pakistan seems to have been affected due to El Nino south oscillation, Pacific decadal oscillation, or Atlantic multi-decadal oscillations.

The article "Recent global warming as a proximate cause of deforestation and forest degradation in northern Pakistan" was retracted in 2022. Reasons: compromised peer review; a conflict of interest; concerns about the authorship.

## Introduction

Drought adversely affects every part of the globe and has a significant impact on the ecosystem good and services [1, 2]. The global percentage of dry areas has increased by about 1.74% per decade from 1950 to 2008 [3]. The increasing occurrence of climate extremes has been noticed with current global warming that had several biophysical impacts worldwide. For instance, the extreme drought spell of 2001–2003 reduced the yield production over 80% in Pakistan and adjacent areas. In the recent past, many drought events such as the 1971 drought also have had disastrous impact on the economy, society, and the ecology of Pakistan. However, the current rate of deforestation is equally a concern for global warming and climatic changes across the globe [4–6]. Similarly, the rate of forest defoliation, forest degradation, and tree mortalities has also increased due to climate changes. It is believed that more than 80% of the original forest cover has been lost, with the remainder distributed in a fragmented agriculture-forest mosaic [7, 8].

Deforestation affects the dynamics of climate system, disturbing hydrological cycles, and causes biodiversity loss both at the regional and global scales [9] when climate change happens, it also accelerates deforestation and degradation. The most pronounced effects of global warming are drought events inducing tree mortality, stunted tree growth, and increasing the chances of forest fire and windstorms [10]. Among them, drought is a primary direct disturbance agent that increases deforestation and affects forest productivity at both regional and global scales [11–16]. This has been documented in Europe, South America, Africa, Australia and the whole of Asia.

Pakistan is an arid and semi-arid country whose economy is largely based on agriculture. The northern forest of Pakistan is considered a good biodiversity hotspot. Unfortunately, this forest is more prone to droughts, windstorms, floods, and forest fires. In the northern hemisphere, forests are more susceptible to natural calamities such as insect outbreak, forest fires, flooding, and soil erosions [17–19]. These hazards have caused widespread damages and losses in the country [20–26]. Forest policymakers often limit themselves around timber management and less attention has been paid to potential threats such as global warming and tree mortality [27–31].

A growing number of studies show that the ongoing climate change will likely accelerate forest degradation but very less work has been done for northern Pakistan so far. The past climatic records are seriously lacking while climate extreme events are barely documented. The instrumental data is not enough to be used in developing climate scenarios. Instrumental data precisely gauge the climatic variability; however. it is hardly available for more than 150 years in the global context while slightly over forty to fifty years in Pakistan with an uneven spatial distribution. Hence instrumental data cannot serve the purpose of assessing the full spectrum of the climatic fluctuation and precisely gauge the amplitude of global warming on a longer timescale.

The article "Recent global warming as a proximate cause of deforestation and forest degradation in northern Pakistan" was retracted in 2022. Reasons: compromised peer review; a conflict of interest; concerns about the authorship.

Palaeoclimatological studies are often based on tree ring growth to extend the climate record back in time because of its linear and constant relationship with tree ring growth and climate limiting variables [31–34]. Tree biomass and certain species are very sensitive to evapotranspiration, soil and air temperatures, air humidity, and soil moisture [34, 35]. This relationship also provides an opportunity to better project how the ongoing climate change will affect tree growth in the future. Up to some extent, it can also project how the climate trend will be in the future. Tree rings are best viable source, documenting every climate-driven event, and provide precisely datable high-resolution climate proxies. Based on tree ring climatic reconstructions, we can extend the existing climatic records for various timescales. However, the response of different species is not uniform and the site qualities, microclimatic conditions have also some pronounced effect on tree growth [36, 37]. The growth rate of tree rings is also different in different time periods; therefore, we have targeted the summer temperature for our reconstruction.

More recently. the expected damages of climate extremes are focused in documenting but recording the magnitude of spatiotemporal impact of climate change due to deforestation and drought is one of the grand emerging challenges [38, 39]. Drought indices are an attempt to examine the magnitude of drought severity along with their effect on the society. The impact of precipitation and temperature on tree growth is little more complex, and there are no perfect techniques to separate precipitation signals from temperature ones. However, scPDSI has been the preferred metric for reconstructing past climatic variation based on temperature and precipitation sensitivity coupled with general soil water holding capacity.

Deforestation and degradation are the main cause of substantial carbon emission in tropical forest, which has global Impacts on the balance and sustainability of the global climate system [40–45]. Forest fires in tropical forest is basically due to extreme drought, these disturbances are the major threats to the worldwide forest ecosystems [17, 46]. In the Amazon region several research studies are carried out to find the impacts of these disturbances [17, 47]. Less attentions are given to the world’s most fragmented West African tropical forests, so this region needs more research work because it is prone to drought, historically drought has a large-scale impact on the socio economic, environmental and ecological conditions [48–52]. Forest microclimates and foster rapid forest degradation is changed rapidly in these fragmented forests because they are vulnerable to forest fire and drought [53, 54]. As a result, forest resilience is compromised due to warmer and drier climates [17] and ultimately these western African tropical forest are endangered. Furthermore, forest degradation and loss are due to the positive response in the forest fire regime, climate change and land use change [46, 55–57].

The article "Recent global warming as a proximate cause of deforestation and forest degradation in northern Pakistan" was retracted in 2022. Reasons: compromised peer review; a conflict of interest; concerns about the authorship.

Increase in human population, economies and land use system the forest ecosystem is rapidly and directly changed. But the ongoing climate change on the forest is very less evident. World scientific community has acknowledged the role of greenhouse gases emission in raising the global mean temperature (about 0.5 8C since 1970) hydrological cycle is also changed [58, 59] also the spread of tropical belt on earth surface [60, 61].

Total forest area of Pakistan hardly reaching to 5.%, though this percentage of forest are consistently under huge pressure of degradation and deforestation [62, 63]. Forest cover area in the world is 30.3% [64, 65], which is very low and not enough. Pakistan has the lowest forest area as compared to other countries in south Asia like Sri Lanka (30%), Bhutan (68%), and India (22.8%) Nepal (25.4%), and Bangladesh (6.7%) [64]. From 1990 to 2010, Pakistan has face the rapid deforestation in 170,684 ha of forest area. [66]. All over the country, Khyber Pakhtunkhwa (KPK) province is the biggest victim (40%) and Gilgit-Baltistan (15.8%). In Pakistan the Himalayan forest ranges play an important role in the livelihood of local community as well as low region areas around these mountains [67]. Local communities derives different kind of products from these forests like wood, medicinal plants, fruits, and vegetables as well as fodder [68, 69]. in Himalayan region the forest is used for many purposes like medicinal plants, aromatic plants, timber, construction, honey and bee keeping, fuel wood and grazing. [70]. A vast majority of households in Gilgit-Baltistan are dependent on forests for their livelihood [62, 71, 72]. Although there is a great development in agriculture and, in developing counties forest resources still play a vital role in rural livelihood and security among the local communities [32–34, 73]. World’s highest mountain peaks are located in these Himalaya, Hindu Kush and Karakorum ranges of Pakistan, including the most famous and important K2, which is the world’s second tallest mountain at 8,611m above sea level [35, 36].

The article "Recent global warming as a proximate cause of deforestation and forest degradation in northern Pakistan" was retracted in 2022. Reasons: compromised peer review; a conflict of interest; concerns about the authorship.

Furthermore, Pakistan is facing some of biggest environmental threats, such as flooding, biodiversity mitigation, decrease in soil fertility, land productivity decrease, soil and water erosion, salinity and loss of vegetation., increasing overgrazing, etc. water scarcity also causing drought in local areas of Pakistan, land production is also reduced because of mismanagement and planning, poverty in Pakistan is due to above mentioned reasons.

Pakistan has the second highest deforestation rate in Asia. Which is a remanding situation [37, 74]. The environment and economy of the Himalayan plains are badly affected by the change in hydrological cycles, floods, desertification and siltation. The losses in environmental conditions are going beyond these Himalayan mountain regions [74, 75]. Contamination also causes morbidity and mortality due to land degradation glitches; overexploitation of fertilizers, pesticides and misuse of natural resources also causes the decrease in soil productivity and spoil drinking water quality. In this manner, here we going to show morbidity and mortality influenced employment methodologies and reinforced reliance on natural assets. Generally, the minor regardless developing group of review proof to critical connections between household’s, mortality and indigenous habitat interceded through business adapting techniques of local communities. The fundamental presumption of this structure is that natural resources have huge mitigative impacts when family units are associated with morbidity and mortality through giving extra demand of pay and significant products that may somehow or another be bought. natural resources is in critical interest during the time of drought, starvation and natural disaster events [76]. Mortality will apply heavier burden on family income under the condition that a large portion of the provincial families in Pakistan have just lived in villages [77].

This study based on *Q*. *incana* tree ring record will deepen our understanding about the past climatic variabilities, the interconnection of deforestation with climate change along with current rate of tree die-off, and spatiotemporal linkages of drought. This study will also formulate a policy under which immediate actions need to be taken.

The article "Recent global warming as a proximate cause of deforestation and forest degradation in northern Pakistan" was retracted in 2022. Reasons: compromised peer review; a conflict of interest; concerns about the authorship.

## Material and method

### Study area

The study sites fall in the northern region, extending up to 3500 km from north to south (°36′18.1″ N, 37°52′29.1″ E; weather station code 41508.5; Fig 1). The precipitation data was collected from the nearby stations. This area is mostly under the shadows to monsoon rainfall, with hot summers, cold winters, and moderate springs and autumns. The precipitation here is received in the form of snow and rain and during March–April see the heaviest rain while June–July are the hottest months (Fig 2).

**Fig 1:** Illustrating the study area map on the northern Pakistan.

**Fig 2:** Monthly maximum, mean, minimum temperature (^0^C) and total precipitation (mm) in the northern Pakistan.

The forest soil is mostly acid to loamy, having less water holding capacity. The Alpine Forest is mostly composed of *Primula elliptica*, *Allium oreoprasum*, *Pulsatilla wallichiana*, *Saussurea simpsoniana* and *Salix karelinii*. The correlation of deforestation and forest degradation with Palmer drought sensitivity index (PDSI) was analyzed to understand the role of ongoing climatic changes on the structure and composition of forest.

The PDSI value was downloaded from KNMI (https://climexp.knmi.nl/get_index.cgi) with the nearest grid point. The precipitation and rainfall data were received from the Gilgit-Baltistan Province in Pakistan.

### Tree rings collection and chronology development

The tree ring cores were received form *Quercous incana*, which is considered to be the most sensitive specie to drought and climate change in the region. Three different sites were chosen for data collection and 30 cores (total 90) from each site were collected.

### Sampling

The tree cores were dried, glued, mounted, and polished. Then it was cross dated by visual growth pattern matching. All the poor qualities tree cores (e.g., fragmented, rotten, and not cross-datable) were discarded from further analyses. COFECHA was used to cross date the series. The final chronologies were developed with the *R* dplr program. The raw ring width series were standardized to elicit biological growth and the standardization was carried out in two steps. A cubic smoothing spline with a 50% frequency-response cutoff equal to 67% of the series length. All detrended series were averaged to chronologies by computing the bi weight robust mean in order to reduce the influence of outliers. The standard protocol used by [78] was followed to get valid results. Expressed population signal (EPS) was used to test the sensitivity of tree response to drought (Table 1).

The article "Recent global warming as a proximate cause of deforestation and forest degradation in northern Pakistan" was retracted in 2022. Reasons: compromised peer review; a conflict of interest; concerns about the authorship.

**Table 1:** Dendrochronological statistics of the *Q*.*incanna* of three study sites.

Site	No trees (cores)	Mean tree ring width ± SD (mm)	ACI	MS	Rbar	EPS
2	65	1.6±0.78	0.45	0.26	0.62	0.85

Variables” abbreviation: Mean Sensitivity (MS), first-order autocorrelation of tree-ring width (ACI), residual ring-width indices Rbar, Expressed Population Signal (EPS).

### Statistical analysis

For the purpose of drought reconstruction, we calculated the Pearson correlation coefficient between the tree ring chronology scPDSI, precipitation over the common period of 1960–2016. Tree-clam R program was used to calculate the correlation coefficient. Among all climate variables, PDSI was found to have the highest correlation with *Q*. *Incana* stand (Fig 4). Signal strength of the site chronologies was assessed by the mean inter-series correlation (Rbar) and with EPS [79]. A standard level of 0.85 in EPS was used to indicate a satisfactory quality of a chronology. The multi-taper method was used to assess the spatial and temporal changes in the region while linear regression was used to predict the response of tree ring width to drought.

## Results

### Characteristics of tree ring chronology

The statistical analysis of 65 tree cores showed that *Q*. *Incana* backed to 264 years had a sufficient common signal and response that might be suitable for dendroclimatic study (Fig 3). The mean series intercorrelation was recorded 0.456. Our results shows that the value of MS (0.26) and EPS (0.85) are considered as a satisfactory response to climatic change [78]. Based on the threshold value for EPS (5 cores >0.85) the period going back to 1700 from 2014 has been selected for the chronology while values lower than this have been truncated.

**Fig 3:** (A) The tree-ring width chronology 1700 to 2019 of site one. (B) Showing the tree-ring width of second site. The gray color represents the sample depth.

### Correlation of chronology with PDSI

Fig 4 shows that tree ring width has a significant (*p*<0.05) correlation with scPDSI for all months, however, May-June recorded the highest value. Further screening for previous year over the current year’s months, the results showed that previous June-October were also critical for the tree ring width. The growth had declined in dry years and narrow rings were noted. The hot drought June-October of the previous year also badly affected the tree growth. The role of precipitation was found significantly (*p*<0.05) positive for the October of the previous year and for the February-May of the current year; only negative response was found for the September of the previous year.

**Fig 4:** Showing Person correlation coefficients between tree-ring index of *Q*. *incanna* monthly total precipitation and PDSI (1960–2016). Significant correlations (*p*<0.05) are denoted by asterisks.

The article "Recent global warming as a proximate cause of deforestation and forest degradation in northern Pakistan" was retracted in 2022. Reasons: compromised peer review; a conflict of interest; concerns about the authorship.

This result exhibits that warm September with low precipitation is most favorable for tree growth. Similarly, the positive precipitation exhibited that good precipitation is the primary requirement for *Q*. *Incana*. The linear regression model showed *F* = 47, *P*<0.001, adjusted *R*^2^ = 0.44, *r* = 0.67, which are significant.


Y=4.53x‐4.97

Here, *Y* shows the results for PDSI and *x* shows the tree ring index. The slope shows the existence of drought signal in the region. Three wet periods were found in 1980–2010, 1812–1836, and 1754–1760 while three dry periods were found in 1896–1922, 1864–1876, and 1784–1788 Figs 5 and 6.

**Fig 5:** Illustrating the relationship of tree-ring width measurement with observed scPDSI for the period of 1960–2014.

**Fig 6:** May-August scPDSI reconstruction for northern area in Pakistan, for the period 1750–2014 along with 11-year low pass filter, mean of the long-term reconstruction illustrated by light pink color of mean ± .5 standard deviation.

The wavelet analysis revealed drought variability at the periodicities of 2.2–2.5, 3.3, 3–4, 16.7, 16.8, and 68–78.8 years. The analysis using multi taper method showed that the variation of drought in northern Pakistan was affected due to El Niño south oscillation, Pacific decadal oscillation and Atlantic multi-decadal oscillations (Figs 7 and 8).

**Fig 7:** The MTM spectrum analysis of the scPDSI from 1700 to 2019. Red and blue line represents the 95% and 99% confidence level, respectively.

**Fig 8:** The wavelet transform from Mar-Feb during 1700 to 2019.

## Discussion

During drought events, the rate of evaporation increases and soil moisture decreases which creates water stress. As a result of water stress, the rate of cell division declines and narrow rings are formed and forest productivity is reduced [39, 40]. Narrow rings and tree mortality rate were used to find out the impacts of climatic changes over forest degradation and tree mortality. It has been concluded that *Q*. *incana* tree ring width was sufficiently limited by drought. The formation of narrow rings and increased tree mortality shows that these species are very sensitive to drought.

Keeping in mind the results, the ongoing climatic changes are supposed to be the immediate cause of deforestation and forest degradation. Beside other factors, increased rates of forest degradation and tree mortality are closely associated with climatic changes. Global warming increases extreme drought events that lead to deforestation and forest degradation at an alarming rate [43]. Forest polices and forest management policies in Pakistan are focusing on forest products while neglecting the potential threats that degrade the forest.

The article "Recent global warming as a proximate cause of deforestation and forest degradation in northern Pakistan" was retracted in 2022. Reasons: compromised peer review; a conflict of interest; concerns about the authorship.

The 1980–2010, 1812–1836, and 1754–1760 dry periods and the 1896–1922, 1864–1876, and 1784–1788 wet periods were coherent with other reconstructions for the surrounding areas [3, 80]. The second most severe drought years featured in our chronology before 1999–2001 was 1970–1971 drought that extended to Tajikistan, India [81, 82] and China [83]. To investigate the common large-scale temperature signals and the representative nature of our reconstruction series, we compared our new record with other reconstructions from the surrounding areas. Our dry and wet periods were close to the dry and wet periods of Treydte et al. (2006). The dry and wet episodes that were prominent in our series were also well matched with the simultaneous dry and wet periods reported by Ahmad et al. (2020). In general, the overall agreement between our reconstruction and other reconstructions suggests that our series is reliable over the past millennium.

Long-term variability indicates that this climate is mostly controlled by mid-latitude westerlies, large-scale wet little Ice Age and western disturbances. The Himalaya region gets precipitation from monsoon rains and western disturbance in the form of rainwater and snow. The 1970–1971 winter received little snow monsoon rainfall that led to severe drought, food shortage, loss of cattle, and environmental problems. It is assumed that the variability in North Atlantic Oscillation and El Nino Southern Oscillation ultimately lead to the failure of monsoon and western disturbance [81, 84, 85]. The dynamic weakening of monsoon probably happened due to the variability in different circulation patterns [86].

The recurring nature of drought and duration of drought will intensify the rate of deforestation and degradation in the near future. Our results are in agreement with the results of [11, 12, 16, 87]. The short-term drought mainly happens due to El-Nino Southern Oscillation; however, long-term drought is caused by large-scale oceanic viabilities such as Atlantic Multidecadal Oscillation, and Pacific Decadal Oscillation. Such climatic variabilities lead to loss of biodiversity and forest degradation as factor of global warming. Due to habitat destruction, most of the wildlife and plants species are on the verge of extinction. The most intense drought, with an intensity of early 1970s, whereas the drought in the mid-2000s experienced the worst peak was also found in our reconstruction [88]. This particular drought was due to an El Niño event, which started to develop in the Pacific ocean in 1997 [89]. These kinds of drought caused severe shortage of water, where hundreds of cattle and livestock perished because of water stress. Our reconstruction also showing that tree-die due to drought enhancing forest fire causing deforestation and forest degradation during above mentioned drought periods. Terrestrial ecosystem is nearly diminishing while species transformation and vegetation is noticed. Change in the climate influences the common pattern of precipitation that leads to unexpected flood, thunderstorms, erosions, famines, and drought events. Even destabilization and migration of civilization has happened in the region due to changing climatic.

The article "Recent global warming as a proximate cause of deforestation and forest degradation in northern Pakistan" was retracted in 2022. Reasons: compromised peer review; a conflict of interest; concerns about the authorship.

These climatic changes increase water stress that might reduce tree growth, degrading the forest quality, and more recently tree mortality. Our results are in agreement with the findings of pre-existing studies [90–92].

Forest fire was also found as the potential cause of drought. Dry vegetation makes the forest more prone to fires. When moisture is dried during droughts, the leaves of *Q*. *Incana* ignite very easily and cause ground fire [39]. The local people were found using the leaves of *Q*. *Incana* for fire activities.

Despite climatic variability, the high dependency on forest resources make the condition worse in the northern region. There are few alternative sources available for fuel and building construction. The use of charcoal cause pollution and add to greenhouse gases while the climatic changes cause forest degradation. In addition, increasing population, level of poverty, low per capita income, and less job opportunities are indirect plausible reasons of deforestation.

There is no clear indicator to measure the role of climatic changes including deforestation and forest degradation on a spatiotemporal scale, but it is was found that the climatic changes are closely associated with the current rate of deforestation and forest degradation in the region. This study suggests a more robust mechanism to study the dynamics of deforestation and forest degradation in the light of ongoing climate changes and indexing the casual links because dry temperate forest are particularly prone to natural disturbance and climatic changes.

## Conclusion

Tree ring chronologies of *Q*. *Incana* was developed. Based on the chronology from *Q*. *Incana*, May–July significant correlation (*r* = 0.59, *p* < 0.01) was applied to reconstruct scPDSI for 264 years with reliable coverage from 1750 to 2014. This reconstruction was found coherence after putting with other dendroclimatic study. Wet periods were found during 1980–2010, 1812–1836, and 1754–1760, while dry periods were found during 1896–1922, 1864–1876, and 1784–1788. Our reconstruction explains 39.8% of the scPDSI variance. Wavelet analysis revealed drought variability at periodicities of 2.2–2.5, 3.3, 3–4, 16.7, 16.8, and 68–78.8 years. Our study finding highlight the high susceptibility of droughts along with deforestation and degradation for *Q*. *Incana* in the northern region of Pakistan and underscore the need to deepen our understanding of the short- and long-term growth-responses of trees to drought.
